The article "Correlation between Serum ApoC III and Galectin-3 Levels and Maternal and Neonatal Adverse Outcomes in Gestational Diabetes Mellitus Patients" was retracted in 2024. Reasons: signs of a paper mill; suspected computer-generated content; unreliable results or conclusions; lack of ethics approval or compliance.

# Correlation between Serum ApoC III and Galectin-3 Levels and Maternal and Neonatal Adverse Outcomes in Gestational Diabetes Mellitus Patients

**DOI:** 10.1155/2022/5089529

**Published:** 2022-09-22

**Authors:** Tingting Tang, Liguang Chen

**Affiliations:** Department of Gynaecology and Obstetrics, Quanzhou First Hospital, Fujian Medical University, Quanzhou, Fujian 362000, China

## Abstract

**Objective:**

The correlation between serum ApoC III and galectin-3 levels and adverse maternal and infant outcomes in GDM patients was analyzed.

**Methods:**

A total of 97 GDM patients admitted to our hospital from January 2019 to June 2021 were selected and divided into a good group and a poor group according to the pregnancy outcomes, ApoC III in blood of subjects was detected by immunoturbidimetry, and galectin-3 level was detected by enzyme-linked immunosorbent assay. Spearman correlation test was used to analyze the correlation between ApoC III and galectin-3 levels and pregnancy outcomes in patients with GDM, and ROC curves were drawn to analyze the value of each index alone and in combination to predict pregnancy outcomes in patients with GDM.

**Results:**

The levels of ApoC III and galectin-3 in the blood of the patients in the bad group were significantly higher than those in the good group, and the difference was statistically significant (*t* = 11.231, 14.965, *P* < 0.05). The levels of ApoC III and galectin-3 in the blood of GDM patients were significantly positively correlated with adverse pregnancy outcomes, and there was a statistical significance (*r* = 0.754 and *r* = 0.698, *P* < 0.05). The combined application of ApoC III and galectin-3 levels in GDM patients' blood to predict the adverse outcome of pregnancy was Log *P* = 0.623,^*∗*^ ApoC III+0.605^*∗*^ galectin-3. The sensitivity, specificity, and AUC of combined application of ApoC III and galectin-3 for predicting adverse pregnancy outcomes in GDM patients were all greater than 90%, and AUC>0.90. The combined application in predicting adverse pregnancy outcomes were higher than those of the individual indicators, and the difference was statistically significant (*P* < 0.05).

**Conclusion:**

The levels of ApoC III and galectin-3 in the blood of GDM patients with adverse pregnancy outcomes were significantly increased, and the detection of ApoC III and galectin-3 could effectively improve the value of predicting adverse pregnancy in GDM.

## 1. Introduction

Gestational diabetes mellitus (GDM) is a common pregnancy complication in women [1]. The results of the study show that the prevalence of GDM in some parts of our country shows an obvious upward trend year by year, which has a serious adverse impact on maternal and child care [2]. GDM may lead to maternal complications such as preeclampsia, spontaneous abortion, and other complications and neonatal complications such as macrosomia, hypoglycemia, deformed infants, and other neonatal complications. At present, the clinical pathogenesis of GDM is not fully understood, but some scholars have pointed out that the occurrence and development of GDM is similar to the pathological basis of type 2 diabetes. [3]. In recent years, studies have found that adipokines are involved in the progression of GDM and are involved in abnormal secretion of adipokines, resulting in abnormal adipose tissue hyperplasia and distribution [4]. Apolipoprotein CIII (ApoC III) is the main apolipoprotein of very low density lipoprotein cholesterol, which has the function of inhibiting the apoE receptor and lipoprotein lipase of liver cell membrane and plays an important role in the regulation of adipose tissue [5]. Galectin-3 is an important *β*-galactoside binding protein in the body and plays a very important role in the occurrence and development of insulin resistance [6]. However, the relationship between ApoC III and galectin-3 levels and adverse maternal and infant outcomes in GDM patients has not been reported yet. Therefore, this study selected GDM patients as the research subjects to analyze the correlation between serum ApoC III and galectin-3 levels and adverse maternal and infant outcomes in GDM patients.

The article "Correlation between Serum ApoC III and Galectin-3 Levels and Maternal and Neonatal Adverse Outcomes in Gestational Diabetes Mellitus Patients" was retracted in 2024. Reasons: signs of a paper mill; suspected computer-generated content; unreliable results or conclusions; lack of ethics approval or compliance.

## 2. Materials and Methods

### 2.1. Research Objects

A total of 97 GDM patients admitted to our hospital from January 2019 to June 2021 were selected as the research subjects, and all patients were divided into a good group and a poor group according to the pregnancy outcomes. There were 64 cases in the good group (age: (28.19 ± 4.32) years, gestational age: (39.28 ± 1.83) weeks, and body weight: (25.38 ± 2.12) kg/m2) and 33 patients in the adverse group, with an age of (28.94 ± 4.71) years, a gestational age of (39.41 ± 1.92) weeks, and a body weight of (25.45 ± 2.37) kg/m2. Inclusion criteria were as follows: (1) meet the diagnostic criteria in the Recommended Guidelines for Clinical Diagnosis and Treatment of Pregnancy Complicated Diabetes (Draft) [7]; (2) GDM confirmed by clinical manifestations combined with laboratory tests; (3) no blood sugar control before admission treatment; (4) prepregnancy diabetes; and (5) singleton pregnancy. Exclusion criteria were as follows: (1) combined with other pregnancy complications such as gestational hypertension; (2) combined with endocrine diseases such as hyperthyroidism and hypothyroidism; (3) polycystic ovary syndrome; (4) combined with severe brain, kidney, liver, heart, lung, and other diseases; and (5) combined with severe trauma or infection. There was no significant difference in general data between the two groups (*P* > 0.05).

The article "Correlation between Serum ApoC III and Galectin-3 Levels and Maternal and Neonatal Adverse Outcomes in Gestational Diabetes Mellitus Patients" was retracted in 2024. Reasons: signs of a paper mill; suspected computer-generated content; unreliable results or conclusions; lack of ethics approval or compliance.

### 2.2. Instruments and Reagents

Low-speed centrifuge (Beckman Avanti JXN-30/26) and Automatic biochemical analyzer (Beckman 5830) were provided by our hospital. Galectin-3 ELISA kit was purchased from Shanghai Xitang Biotech Co., Ltd.

## 3. Methods

After the subjects were enrolled, fasting venous blood was collected, the speed was 3000 r/min, and the serum was collected by centrifugation at four degrees for 10 min. The level of ApoC III in the blood of subjects was detected by Beckman 5830 automatic biochemical analyzer. Galectin-3 levels were detected by enzyme-linked immunosorbent assay, all operations were carried out in strict accordance with the kit instructions, and the quality control and detection were carried out in accordance with the standard operating procedures of the instrument.

### 3.1. Statistical Methods

SPSS 20.0 was used for statistical analysis, and the count and measurement data were expressed by percentage and mean ± standard deviation, and then the chi-square test and LSD-t test were used to analyze the differences of count data and measurement data between groups. Spearman correlation test was used to analyze the correlation between ApoC III and galectin-3 levels and pregnancy outcomes in GDM patients. The logistic regression model was used to analyze the combined model of ApoC III and galectin-3 for predicting pregnancy outcome in GDM patients. ROC curves were then drawn to analyze the value of each index alone and in combination to predict the pregnancy outcome of GDM patients. *P* < 0.05 indicates that the difference is statistically significant.

## 4. Results

### 4.1. Test Results of ApoC III and Galectin-3 Levels in Blood of Subjects

The results of this study showed that the levels of ApoC III and galectin-3 in the blood of the patients in the poor group were significantly higher than those in the good group, and the difference was statistically significant (*P* < 0.05), as shown in Table 1.

### 4.2. The Correlation between ApoC III and Galectin-3 in Subjects' Blood and Pregnancy Outcome

The results of this study showed that the levels of ApoC III and galectin-3 in the blood of GDM patients were significantly positively correlated with adverse pregnancy outcomes (*r* = 0.754 and *r* = 0.698), and there was a statistically significant difference (*P* < 0.05).

### 4.3. ApoC III and Galectin-3 Combined Model for Predicting Pregnancy Outcomes in GDM Patients

. The results of this group showed that the ApoC III level in the blood of GDM patients to predict the adverse pregnancy outcome model of patients is *P* = 0.623,^*∗*^ The Galectin-3 level to predict the adverse pregnancy outcome model of patients is ApoC III+0.605^*∗*^, as shown in Table 2.

The article "Correlation between Serum ApoC III and Galectin-3 Levels and Maternal and Neonatal Adverse Outcomes in Gestational Diabetes Mellitus Patients" was retracted in 2024. Reasons: signs of a paper mill; suspected computer-generated content; unreliable results or conclusions; lack of ethics approval or compliance.

### 4.4. The Value of ApoC III and Galectin-3 in Predicting Pregnancy Outcomes in GDM Patients

The results of this study showed that the combined application of ApoC III and galectin-3 had sensitivity and specificity greater than 90% and AUC >0.90 in predicting adverse pregnancy outcomes in patients with GDM. The sensitivity, specificity, and AUC of the combined application in predicting adverse pregnancy outcomes were higher than those of the individual indicators, and the difference was statistically significant (*P* < 0.05), as shown in Table 3 and Figure 1.

## 5. Discussion

GDM is one of the common pregnancy complications. Some studies have shown that pregnant women with GDM have premature rupture of membranes, termination of pregnancy, polyhydramnios, gestational hypertension, and postpartum hemorrhage. The incidence of infant asphyxia, macrosomia, premature infant, and neonatal pneumonia was higher than that of normal pregnancy [8]. GDM usually has no obvious symptoms in the first trimester, and the fasting blood glucose level is basically normal in clinical screening, so the clinical missed diagnosis rate is high. GDM has a greater impact on both mother and baby, and effective evaluation and treatment can improve the clinical outcomes of patients. Pregnancy outcomes are of great significance [9]. Research results show that obesity-induced lipotoxicity plays a very important role in the occurrence and development of GDM. The proliferation of adipocytes can be achieved by detecting and observing adipokines and can be used to analyze the changes of GDM disease [10]. In addition, previous studies have pointed out that GDM can be predicted by detecting inflammatory factors and glucose metabolism indicators related to type 2 diabetes, which suggests that the occurrence and development of type 2 diabetes has many similarities with GDM, but the relationship between inflammatory factors, lipid metabolism related indicators, and pregnancy outcomes of GDM patients has rarely been reported. The relationship with pregnancy outcomes in GDM patients is still rarely reported [11].

Studies have pointed out that a large number of bioactive factors such as leptin and ApoC III are synthesized and secreted by adipocytes and play a very important role in the occurrence and development of insulin resistance [12]. ApoC III is a diabetes-causing factor that has gradually attracted widespread attention in recent years, and it is of great significance to actively control the level of ApoC III in the process of slowing down the progression of diabetes. ApoC III is a potent direct modulator of established cardiovascular disease risk factors: plasma triglycerides and inflammation. Recent findings show that changes in ApoC III levels are directly associated with changes in directing the atherogenicity of HDL, intestinal dietary triglyceride trafficking, and modulating pancreatic *β*-cell survival. The combination of these roles makes ApoC III an important therapeutic target for the management and prevention of diabetes. ApoC III plays a role in regulating body weight, food intake, and energy metabolism in the body and plays an important role in anti-inflammatory response, anti-intimal hyperplasia after injury, and anti-atherosclerosis [13]. Galectin-3 is synthesized and secreted by a variety of immune cells in the body such as macrophages. Galectin-3 (Gal-3) regulates basic cellular functions such as cell-cell and cell-matrix interactions, growth, proliferation, differentiation, and inflammation. It is not surprising that this protein is involved in the pathogenesis of many relevant human diseases, including cancer, fibrosis, chronic inflammation, and scarring affecting many different tissues. It can bind to insulin receptors in insulin target organs such as adipocytes and muscles to regulate insulin [14].

The article "Correlation between Serum ApoC III and Galectin-3 Levels and Maternal and Neonatal Adverse Outcomes in Gestational Diabetes Mellitus Patients" was retracted in 2024. Reasons: signs of a paper mill; suspected computer-generated content; unreliable results or conclusions; lack of ethics approval or compliance.

The results of this study showed that the levels of ApoC III and galectin-3 in the blood of the patients in the poor group were significantly higher than those in the good group. There was a significant positive correlation with adverse pregnancy outcomes of patients. Further exploration of ApoC III and galectin-3 in predicting pregnancy outcomes showed that the combined application of ApoC III and galectin-3 had sensitivity and specificity greater than 90% in predicting adverse pregnancy outcomes in patients with GDM, and AUC was greater than 0.90. The sensitivity, specificity, and AUC of the outcome were all higher than those of each indicator alone. The analysis shows that the levels of ApoC III and galectin-3 can effectively evaluate the lipid metabolism and inflammatory state in GDM patients. With the increase of ApoC III and galectin-3 levels, it indicates that the abnormal state of lipid metabolism and inflammation in patients is aggravated, accompanied by the appearance of pancreatic islet cells. Abnormal function aggravates, and the phenomenon of insulin resistance increases. It can lead to aggravation of the patient's condition and may lead to the occurrence of adverse pregnancy outcomes. Through the combined detection and analysis of ApoC III and galectin-3 levels, the lipid metabolism and inflammatory state in GDM patients can be deeply studied and analyzed, so it can effectively improve the value of predicting the pregnancy outcome of GDM patients. Insulin resistance in diabetes is strongly associated with chronic inflammation and obesity. Insulin target tissue is affected by inflammatory mediators and undergoes pathological changes that lead to the onset and development of insulin resistance. The high expression of ApoC III may lead to the high expression of blood lipids in the body, induce apoptosis of islet *β* cells, and may aggravate abnormal blood glucose metabolism in patients. Galectin-3 can effectively inhibit insulin secretion, block insulin signaling pathway, regulate chemotaxis such as macrophages and induce the migration of macrophages to insulin target tissues, leading to the synthesis and release of Galectin-3, aggravating insulin resistance, and forming a vicious circle [15].

The article "Correlation between Serum ApoC III and Galectin-3 Levels and Maternal and Neonatal Adverse Outcomes in Gestational Diabetes Mellitus Patients" was retracted in 2024. Reasons: signs of a paper mill; suspected computer-generated content; unreliable results or conclusions; lack of ethics approval or compliance.

In conclusion, the levels of ApoC III and galectin-3 in the blood of GDM patients with adverse pregnancy outcomes were significantly increased, and the detection of ApoC III and galectin-3 could effectively improve the value of predicting adverse pregnancy in GDM. However, the number of clinical samples in this study was small, and no long-term follow-up and follow-up were performed on patients, which needs further research and discussion [16].

## Figures and Tables

**Figure 1:** ROC curve.

**Table 1:** Test results of ApoC III and galectin-3 levels in blood of subjects.

Indexes	Maternal and infant adverse outcome group (*n* = 33)	Good maternal and infant outcome group (*n* = 64)	t	*p*
ApoC III/*μ*g/mL	9.31 ± 1.75	5.59 ± 1.04	11.231	0.001
Galectin-3/*μ*g/mL	35.40 ± 8.34	13.29 ± 2.19	14.966	0.001

**Table 2:** Combined model of ApoC III and galectin-3 for predicting pregnancy outcome in patients with GDM.

Indexes	b	SE	*χ*2	*P*	OR	95% CI	
						Lower limit	Upper limit
ApoC III	0.623	0.229	7.401	0.007	1.865	1.190	2.921
Galectin-3	0.605	0.215	7.918	0.005	1.831	1.202	2.791

**Table 3:** The value of ApoC III and galectin-3 in predicting pregnancy outcome in patients with GDM.

Indexes	Sensitivity	Specificity	AUC	Standard error	*p*	95% CI	
						Lower limit	Upper limit
ApoC III	78.79	85.94	0.785	0.049	0.001	0.690	0.881
Galectin-3	75.76	81.25	0.759	0.054	0.001	0.653	0.864
Joint application	93.94	95.31	0.905	0.040	0.001	0.827	0.984

## Data Availability

The data can be obtained from the corresponding author upon reasonable request.
